# Corticotropin-Releasing Factor Facilitates Epileptiform Activity in the Entorhinal Cortex: Roles of CRF_2_ Receptors and PKA Pathway

**DOI:** 10.1371/journal.pone.0088109

**Published:** 2014-02-04

**Authors:** Lalitha Kurada, Chuanxiu Yang, Saobo Lei

**Affiliations:** Department of Basic Sciences, University of North Dakota, Grand Forks, North Dakota, United States of America; Institut National de la Santé et de la Recherche Médicale (INSERM U901), France

## Abstract

Whereas corticotropin-releasing factor (CRF) has been considered as the most potent epileptogenic neuropeptide in the brain, its action site and underlying mechanisms in epilepsy have not been determined. Here, we found that the entorhinal cortex (EC) expresses high level of CRF and CRF_2_ receptors without expression of CRF_1_ receptors. Bath application of CRF concentration-dependently increased the frequency of picrotoxin (PTX)-induced epileptiform activity recorded from layer III of the EC in entorhinal slices although CRF alone did not elicit epileptiform activity. CRF facilitated the induction of epileptiform activity in the presence of subthreshold concentration of PTX which normally would not elicit epileptiform activity. Bath application of the inhibitor for CRF-binding proteins, CRF6-33, also increased the frequency of PTX-induced epileptiform activity suggesting that endogenously released CRF is involved in epileptogenesis. CRF-induced facilitation of epileptiform activity was mediated via CRF_2_ receptors because pharmacological antagonism and knockout of CRF_2_ receptors blocked the facilitatory effects of CRF on epileptiform activity. Application of the adenylyl cyclase (AC) inhibitors blocked CRF-induced facilitation of epileptiform activity and elevation of intracellular cyclic AMP (cAMP) level by application of the AC activators or phosphodiesterase inhibitor increased the frequency of PTX-induced epileptiform activity, demonstrating that CRF-induced increases in epileptiform activity are mediated by an increase in intracellular cAMP. However, application of selective protein kinase A (PKA) inhibitors reduced, not completely blocked CRF-induced enhancement of epileptiform activity suggesting that PKA is only partially required. Our results provide a novel cellular and molecular mechanism whereby CRF modulates epilepsy.

## Introduction

Epilepsy is a common neurological disorder characterized by excessive excitation of brain regions including the entorhinal cortex (EC), hippocampus and amygdala. The available antiepileptic drugs, while effective, render only ∼40% patients free of seizures after optimal treatment. Furthermore, the antiepileptic drugs have side effects and target a limited number of mechanisms. Therefore, identifying additional mechanisms through which seizures are generated and developing therapeutic strategies targeting these mechanisms are still necessary. Corticotropin-Releasing Factor (CRF) is a peptide of 41 amino acids released from the paraventricular nucleus of the hypothalamus. Whereas the traditional role of CRF is to initiate and regulate the hypothalamic-pituitary-adrenal responses to stress, CRF has increasingly been recognized as a neuromodulator in the extrahypothalamic circuits. CRF immunoreactivity has been detected in the cerebellar cortex [1], locus coeruleus [1], olfactory bulb [2] and the limbic structures including the EC [2], [3], hippocampus [3] and amygdala [4]. The identity of the CRF-containing neurons can be either GABAergic [5] [10] or glutamatergic [6], [7]. CRF interacts with two G protein-coupled receptors (denoted as CRF_1_ and CRF_2_ thereafter) and binds to the CRF-binding protein which buffers the amount of free CRF in the extracellular compartment [8]. CRF_1_ and CRF_2_ receptors display distinct pharmacological profiles and are widely distributed in the extrahypothalamic circuits. CRF_1_ receptors are expressed in pituitary, cerebellar cortex, neocortex, median eminence, and sensory relay nuclei [9], [10], [11] whereas CRF_2_ receptors are localized mostly to subcortical regions including the septum, amygdala, hippocampus and EC [12], [13], [14]. Both CRF_1_ and CRF_2_ receptors are primarily coupled to G_s_ proteins resulting in activation of adenylyl cyclase (AC) and an increase in the level of intracellular cyclic AMP (cAMP) that activates protein kinase A (PKA) [15], [16] although CRF receptors have the ability to interact with other G-protein systems including G_q_, G_i_, G_o_, G_i1/2_, and G_z_ [17] to modulate protein kinase B, protein kinase C, mitogen-activated protein kinases and intracellular Ca^2+^ concentrations in a tissue-specific manner [15], [16]. The biological actions of CRF are likely to be mediated by these CRF receptors and their intracellular signals.

CRF has been implicated in a variety of neurological diseases including the affective disorders and epilepsy [18]. For example, intracerebroventricular injection of CRF induces seizures [19], [20], [21], [22] and seizures alter the expressions of CRF [23], [24], [25], [26], [27], [28], CRF-binding protein [3], [24], [28] and CRF receptors [3], [28], [29] supporting the notion that CRF is the most potent epileptogenic peptide [18]. However, several essential issues regarding the roles of CRF in epilepsy have not been addressed. For example, what is the action site in the brain for the effects of CRF on epilepsy because intracerebroventricular application of CRF can influence almost all the brain regions? Which type of CRF receptors is involved in CRF-mediated facilitation of epilepsy? What are signaling molecules required for CRF-induced facilitation of epilepsy? Since the EC is an important structure involved in epilepsy and mRNA of CRF receptors has been detected in the EC by in situ hybridization [14], we examined the effects of CRF on picrotoxin (PTX)-induced epileptiform activity recorded from entorhinal slices. The PTX-induced seizure model resembles the simple partial and generalized forms of human epilepsy [30], [31], [32]. Our results demonstrate that CRF increases the epileptiform activity induced by PTX via activation of CRF_2_ receptors. CRF-mediated facilitation of epileptiform activity required the functions of AC and cAMP but PKA is partially involved. Our results provide a novel molecular mechanism to explain the roles of CRF in epilepsy.

## Materials and Methods

### Slice preparation

Horizontal brain slices (350 µm) including the EC, subiculum and hippocampus were cut using a vibrating blade microtome (VT1000S; Leica, Wetzlar, Germany) from Sprague-Dawley rats (13- to 18-day-old), wild-type (WT) and CRF_2_ knockout (KO) mice (1 month) as described previously [33], [34], [35], [36]. After being deeply anesthetized with isoflurane, animals were decapitated and their brains were dissected out in ice-cold saline solution that contained (in mM) 130 NaCl, 24 NaHCO_3_, 3.5 KCl, 1.25 NaH_2_PO_4_, 0.5 CaCl_2_, 5.0 MgCl_2_, and 10 glucose, saturated with 95% O_2_ and 5% CO_2_ (pH 7.4). Slices were initially incubated in the above solution at 35°C for 40 min for recovery and then kept at room temperature (∼24°C) until use.

### Recordings of epileptiform activity from entorhinal slices

Slices were bathed in the extracellular solution comprised (in mM) 130 NaCl, 24 NaHCO_3_, 5 KCl, 1.25 NaH_2_PO_4_, 2.5 CaCl_2_, 1.5 MgCl_2_ and 10 glucose, saturated with 95% O_2_ and 5% CO_2_ (pH 7.4). Spontaneous epileptiform activity was induced by including the GABA_A_ receptor blocker PTX (100 µM) in the preceding extracellular solution [37], [38]. An electrode containing the extracellular solution was placed in layer III of the EC to record epileptiform activity. After stable spontaneous epileptiform activity occurred, which usually took ∼20 min, CRF was applied in the bath. The epileptiform events were initially recorded by Clampex 9.2 and subsequently analyzed by Mini Analysis 6.0.1.

### Immunocytochemistry

Procedures for immunocytochemistry were described previously [39], [40], [41], [42], [43]. Briefly, rats (18-day-old) were anaesthetized with pentobarbital sodium (50 mg/kg) and then perfused transcardially with 0.9% NaCl followed by 4% paraformaldehyde in 0.1 M phosphate-buffered saline (PBS). Brains were rapidly removed and postfixed in the same fixative for an additional 2 h. After postfixation, brains were cryoprotected with 30% sucrose in PBS for 12 h and then cut into 20 µm slices in thickness horizontally in a Leica cryostat (CM 3050 S) at −21°C. Slices were washed in 0.1 M PBS and then treated with 0.3% hydrogen peroxide (H_2_O_2_) to quench endogenous peroxidase activity. After being rinsed in 0.1 M PBS containing 1% Triton X-100 and 1.5% normal donkey serum for 30 min, slices were incubated with the primary antibodies (goat anti-CRF antibody, sc-1761; anti-CRF_1_ antibody, sc-12381; anti-CRF_2_ antibody, sc-20550; Santa Cruz Biotechnology Inc.) at a dilution of 1∶100 at 4°C for 12 h. Slices were incubated at room temperature initially with biotinylated donkey anti-goat IgG (ABC Staining System, Santa Cruz Biotechnology Inc.) for 1 h and then with avidin-biocytin complex (ABC Staining System) for 30 min. After each incubation, slices were washed three times for a total of 30 min. Diaminobenzidine (ABC Staining System) was used for a color reaction to detect the positive signals. Finally, slices were mounted on slides, dehydrated through an alcohol range, cleared in xylene and covered with cover-slips. Slides were visualized and photographed with a Leica microscope (DM 4000B). We stained 5–6 nonadjacent sections and each staining was repeated by using 3 rats.

### Western blot

Brain tissues for western blot experiments were taken from 10 rats (18-day-old). For each rat, horizontal brain slices were cut initially and the medial EC region was punched out from the slices under a microscope. The isolated brain region was lysed in tissue protein extraction buffer containing protease inhibitors (Pierce, Rockford, IL). The lysates were centrifuged at 10,000×g for 10 min to remove the insoluble materials and protein concentrations in the supernatant were determined [44]. An equivalent of 40 µg total protein was loaded to each lane. Proteins were separated by 12% SDS–PAGE and transferred to the polyvinylidene difluoride (PVDF, Immobilon-P, Millipore, Billerica, MA) membranes using an electrophoretic transfer system (BioRad, Hercules, CA). Blots were blocked with 5% powdered milk, and then incubated with individual primary antibodies (anti-CRF, anti-CRF_1_ or anti-CRF_2_, 1∶500) overnight at 4°C followed by incubation with the secondary antibody (donkey anti-goat IgG-HRP, 1∶2000) for 1 h at room temperature. Tris-buffered saline with 1% Tween-20 was used to wash the blots 3 times (10 min each) after incubation with both primary and secondary antibodies. Immunoreactive bands were visualized by SuperSignal West Pico Chemiluminescent Substrate (Pierce, Rockford, IL) and detected by a Biospectrum Imagining System (UVP, Upland, CA).

### Data analysis

Data were presented as the means ± S.E.M. For statistical analysis of the effects of CRF on epileptiform activity, the averages of 3–5 min of the frequency of epileptiform activity before and after the application of CRF were compared. CRF concentration-response curves were fitted by the Hill equation: *I*  =  *I*_max_ × {1/[1 + (EC_50_/[ligand])*^n^*]}, where *I*_max_ is the maximum response, EC_50_ is the concentration of ligand producing a half-maximal response, and *n* is the Hill coefficient. Student's paired or unpaired *t* test or analysis of variance (ANOVA) was used for statistical analysis as appropriate; *P* values were reported throughout the text and significance was set as *P*<0.05. N number in the text represents the number of slices examined.

### Animals, ethic statement and chemicals

Sprague-Dawley rats were purchased from Harlan Laboratories. CRF_2_ homozygous KO mice (Stock number: 010842; Strain name: B6; 129-*crhr2^tm1jsp^*/J) and WT mice (from the same colony) were bought from Jackson Laboratories. This study was carried out in strict accordance with the recommendations in the Guide for the Care and Use of Laboratory Animals of the National Institutes of Health. The protocol was approved by the Committee on the Ethics of Animal Experiments of the University of North Dakota (0702-2). All efforts were made to minimize suffering. CRF was purchased from American Peptide Company (Sunnyvale, CA). The following reagents were products of TOCRIS (Ellisville, MO): K41498, astressin 2B, NBI 27914, CP 154526, MDL 12330A, SQ 22536, forskolin, 3,7-dihydro-1-methyl-3-(2-methylpropyl)-1H-purine-2,6-dione (IBMX), KT 5720, Rp-cAMPS. The other chemicals were purchased from Sigma-Aldrich (St. Louis, MO).

## Results

### Expression of CRF and CRF_2_ in the EC

We first examined the expression of CRF and CRF receptors in the EC of rats using immunocytochemistry and western blot. The anatomical location of the EC and the divisions of individual layers in slice of rats were described previously [39], [45]. Strong immunoreactivities for CRF (Fig. 1A, upper panel) and CRF_2_ (Fig. 1C, upper panel) were detected in the EC whereas there was no detectable immunoreactivity for CRF_1_ in the EC (Fig. 1B, upper panel). Western blot demonstrates that a band of ∼20 kDa (Fig. 1A, lower panel) close to the reported molecular mass of CRF [46], [47], [48] and a band of ∼63 kDa (Fig. 1C, lower panel) close to the reported molecular mass of CRF_2_ [49] were detected in the lysate of the EC. The specificities of the antibodies were confirmed by the results that preabsorption of the antibodies with their corresponding blocking peptides blocked the detection of the bands (Fig. 1A and 1C, lower panel right). Whereas the molecular mass of rat brain CRF_1_ was found to be 76–80 kDa [50], [51], there was no conspicuous band within this range (Fig. 1B, lower panel) demonstrating that there is no expression of CRF_1_ in the EC. Together, these data demonstrate that the EC expresses CRF and CRF_2_ with no detectable expression of CRF_1_, consistent with previous results obtained by in situ hybridization [14].

**Figure 1:** The entorhinal neurons expresses CRF and CRF_2_ receptors but not CRF_1_ receptors. **A**, Immunoreactivity for CRF (*upper*) and detection of CRF by western blot (*lower*). *Upper right*: high magnification of the region marked in the left. **B**, Lack of immunoreactivity (*upper*) and protein band (*lower*) for CRF_1_ receptors. **C**, The entorhinal neurons showed immunoreactivity (*upper*) for CRF_2_ receptors and western blot detected a band close to the molecular mass of CRF_2_ receptors in the lysates of the EC (*lower*).

### CRF facilitates epileptiform activity recorded from the EC in horizontal slices

We studied the roles of CRF in epilepsy by recording PTX-induced epileptiform activity from layer III of the EC in horizontal slices. As described previously, stable epileptiform events occurred in ∼20 min after bath perfusion of PTX [38]. We therefore began to record basal epileptiform activity after perfusion of PTX for ∼20 min. In this *in vitro* slice seizure model, application of CRF (0.1 µM) in the perfusion solution significantly increased the frequency of the epileptiform activity (n = 7 slices, *P*<0.001, Fig. 2A_1_ and 2A_2_).

**Figure 2:** CRF increases the frequency of epileptiform activity induced by PTX and facilitates the susceptibility to epilepsy. **A_1_–A_2_**, Bath application of CRF increased the frequency of epileptiform activity recorded from layer III of the EC in horizontal slices. **B_1_–B_2_**, Bath application of CRF augmented the frequency of epileptiform activity recorded from layer III of the EC in “mini slices” for which the hippocampus and other cortices were cut away. **C**, Concentration-response curve of CRF-induced facilitation of epileptiform activity. Numbers in the parentheses were numbers of slices recorded. **D_1_–D_2_**, Bath application of subthreshold concentration of PTX (10 µM) for 30 min failed to induce epileptiform activity whereas co-application of CRF induced robust epileptiform activity. **E_1_–E_3_**, Bath application of CRF6-33, a comparative inhibitor of the CRF-binding protein, significantly increased the frequency of epileptiform activity via activation of CRF_2_ receptors. Pre-application of K41498, a selective CRF_2_ antagonist, blocked CRF6-33-induced increases in the frequency of epileptiform activity.

The above experiments were performed in the horizontal slices containing the EC, hippocampus and other cortices. Whereas the connections among the EC and other brain regions such as the hippocampus are unlikely to be complete after cutting of the slices, we still tested whether the effects of CRF on epileptiform activity were due to the action of CRF on structures other than the EC. We therefore cut the medial EC out under a microscope and recorded PTX-induced epileptiform activity from layer III of the EC in this “mini slice”. As shown in Figure 2B_1_ and 2B_2_, bath application of CRF (0.1 µM) still significantly increased the frequency of the epileptiform activity in the mini slices (n = 8, *P* = 0.001, Fig. 2B_1_–2B_2_) excluding the possibility that the action site of CRF is outside of the EC. Because CRF-induced increase in epileptiform activity recorded from the horizontal slices was statistically indistinguishable from that recorded from the mini slices (*P* = 0.98, two-way ANOVA), we used the horizontal slices for the rest of the experiments simply for the convenience of experiments. The EC_50_ for CRF was measured to be 19.6 nM (Fig. 3C). Because the maximal effect of CRF could be observed at 0.1 µM, we used this concentration of CRF for the rest of experiments. Bath application of the saturated concentration of CRF (0.1 µM) without PTX for 20 min failed to induce epileptiform activity (n = 5 slices, data not shown) suggesting that CRF alone is incapable of inducing epileptiform activity in slices. We then tested whether CRF facilitates the susceptibility of epilepsy. Bath application of the subthreshold concentration of PTX (10 µM) for 30 min did not induce epileptiform activity (Fig. 2D_1_ and 2D_2_) but subsequent co-application of CRF (0.1 µM) induced robust epileptiform activity (Fig. 2D_1_ and 2D_2_) suggesting that CRF increases the susceptibility of epilepsy.

**Figure 3:** CRF facilitates epileptiform activity via activation of CRF_2_ receptors. **A**, Pretreatment of slices with and continuous bath application of K41498, a selective CRF_2_ antagonist, blocked CRF-mediated increases in epileptiform activity. **B**, Pretreatment of slices with and continuous bath application of astressin 2B, another selective CRF_2_ antagonist, blocked CRF-mediated increases in epileptiform activity. **C**, Pretreatment of slices with and continuous bath application of NBI 27914, a selective CRF_1_ antagonist, failed to alter significantly CRF-mediated increases in epileptiform activity. **D**, Pretreatment of slices with and continuous bath application of CP 154526, another selective CRF_1_ antagonist, did not change the facilitatory effect of CRF on epileptiform activity. **E**, Application of CRF increased epileptiform activity in WT mice. **F**, Application of CRF did not induce an increase in epileptiform activity in CRF_2_ KO mice.

The above results suggest that endogenously released CRF may play a role in epileptogenesis. As shown in Fig. 1A, high density of CRF immunoreactivity was detected in the EC. Because it is well-known that the release of neuropeptides requires high neuronal activities, we hypothesized that PTX-induced epileptiform activity may have increased CRF release, which further facilitates the epileptiform activity. We therefore tested this hypothesis by probing the roles of endogenously released CRF in PTX-induced epileptiform activity. Because CRF binds to the CRF-binding protein which buffers the amount of free CRF in the extracellular compartment [8], we superfused slices with CRF6-33 (1 µM), a comparative inhibitor of the CRF-binding protein. This peptide was used successfully to test the endogenous role of CRF in facilitating intracellular Ca^2+^ release in midbrain dopamine neurons [52]. Bath application of CRF6-33 significantly increased the frequency of epileptiform activity induced by PTX (236±39% of control, n = 4, *P* = 0.04, Fig. 2E_1_ and 2E_2_). As would be shown below, CRF-mediated increases in epileptiform activity were mediated by activation of CRF_2_ receptors. Pre-incubation of slices with and continuous bath application of the selective CRF_2_ antagonist, K41498 (0.1 µM), blocked CRF6-33-induced augmentation of epileptiform activity (98±9% of control, n = 5, *P* = 0.82, Fig. 2E_3_). These data together demonstrate that endogenously released CRF facilitates epileptiform activity.

### CRF increases epileptiform activity via activation of CRF_2_ receptors

We next probed the roles of CRF receptors in CRF-mediated facilitation of epileptiform activity. Pretreatment of slices with and continuous bath application of K41498 (0.1 µM), a CRF_2_ antagonist, significantly reduced CRF-induced increases in epileptiform activity (122±10% of control, n = 11 slices, *P*<0.001 vs. CRF alone, Fig. 3A). Application of astressin 2B (0.1 µM), another CRF_2_ antagonist, in the same fashion blocked CRF-induced increases in epileptiform activity (113±9% of control, n = 7, *P* = 0.22 vs. baseline, Fig. 3B). Whereas these data demonstrate the requirement of CRF_2_ receptors, we also examined the roles of CRF_1_ receptors. CRF-induced increases in epileptiform activity were not altered significantly (vs. CRF alone) in slices treated with NBI 27914 (1 µM, n = 8, *P* = 0.78, Fig. 3C) or CP 154526 (1 µM, n = 12, *P* = 0.87, Fig. 3D), two selective CRF_1_ antagonists. We further confirmed the role of CRF_2_ receptors by using CRF_2_ receptor KO mice. Application of CRF (0.1 µM) increased the epileptiform activity in WT mice (n = 14 slices from 4 mice, *P*<0.001, Fig. 3E) but did not facilitate the epileptiform activity in CRF_2_ receptor KO mice (n = 12 slices from 3 mice, *P* = 0.59, Fig. 3F) further confirming the requirement of CRF_2_ receptors.

### Roles of the AC/cAMP/PKA pathway in CRF-induced increases in epileptiform activity

Because CRF_2_ receptors are coupled to AC/cAMP/PKA pathway and there is strong evidence demonstrating that cAMP and PKA signals exert a tonic control of epilepsy [53], [54], [55], [56], [57], [58], we tested the roles of this pathway in CRF-mediated facilitation of epileptiform activity. Slices were pretreated with the selective AC inhibitor MDL 12330A (50 µM) for ∼20 min and the same concentration of MDL 12330A was included in the PTX-containing extracellular solution and applied in the bath before and during the application of CRF. In this condition, bath application of CRF (0.1 µM) did not significantly increase the frequency of the epileptiform activity (n = 11, *P* = 0.14, Fig. 4A). Similarly, application of SQ 22536 (400 µM), another AC inhibitor, in the same fashion also blocked CRF-mediated facilitation of the frequency of epileptiform activity (n = 7, *P* = 0.2, Fig. 4B). These data together indicate that CRF increases epileptiform activity via activation of AC.

**Figure 4:** CRF facilitates epileptiform activity via activation of AC/cAMP/PKA pathway. **A**, Pretreatment of slices with MDL-12330A, a selective AC inhibitor, blocked CRF-mediated increases in epileptiform activity. **B**, Pre-application of SQ-22536, another AC inhibitor, blocked CRF-mediated facilitation of epileptiform activity. **C**, Bath application of forskolin, an AC activator, increased the frequency of epileptiform activity. **D**, Bath application of IBMX, a PDE inhibitor, enhanced the frequency of epileptiform activity. **E**, Pretreatment of slices with KT 5720, a selective PKA inhibitor, partially blocked CRF-mediated enhancement of the frequency of epileptiform activity. **F**, Pretreatment of slices with Rp-cAMPS, another specific PKA inhibitor, partially blocked the facilitatory effect of CRF on epileptiform activity.

Activation of AC increases the generation of cAMP. We next tested whether elevation of cAMP level mimics the effect of CRF. Bath application of forskolin (20 µM), an AC activator, significantly increased the frequency of epileptiform activity (170±12% of control, n = 13, *P*<0.001, Fig. 4C). Moreover, application of IBMX (500 µM), a phosphodiesterase inhibitor to inhibit the degradation of cAMP, also significantly increased the frequency of epileptiform activity (253±23% of control, n = 15, *P*<0.001, Fig. 4D). These data together demonstrate that CRF-induced increases in the frequency of epileptiform activity are related to an increase in intracellular cAMP level.

We next tested the roles of PKA in CRF-induced facilitation of epileptiform activity. Slices were pretreated with the selective PKA inhibitor KT 5720 (1 µM) for ∼20 min and the same concentration of KT 5720 was included in the PTX-containing extracellular solution and applied in the bath before and during the application of CRF. In this condition, bath application of CRF (0.1 µM) induced a statistically smaller increase in the frequency of epileptiform activity (130±8% of control, n = 10, *P* = 0.005 vs. CRF alone, Fig. 4E). Application of Rp-cAMPS (100 µM), another specific PKA inhibitor, in the same fashion also significantly diminished CRF-mediated facilitation of the frequency of epileptiform activity (133±4% of control, n = 9, *P* = 0.004 vs. CRF alone, Fig. 4F). These data together demonstrate that PKA also plays a role in CRF-mediated increase in epileptiform activity.

## Discussion

Our results demonstrate that both CRF protein and CRF_2_ receptors are expressed in the EC suggesting that CRF plays an important role in the EC. Indeed, bath application of CRF to entorhinal slices facilitates PTX-induced epileptiform activity via activation of CRF_2_ receptors. CRF-mediated increases in epileptiform activity require the functions of AC and cAMP but PKA is partially involved in CRF-induced facilitation of epileptiform activity.

Whereas intracerebroventricular injection of CRF induces seizures [19], [20], [21], [22], the action sites of CRF have not been identified. Our results demonstrate that the EC is at least one of the action sites for CRF-induced facilitation of epilepsy because application of CRF to the entorhinal slices robustly increased the frequency of epileptiform activity induced by PTX. The action site of CRF is unlikely to be in brain regions other than the EC because application of CRF to the ‘mini’ slices in which other brain regions except the medial EC were cut off still induces the same level of facilitation of PTX-induced epileptiform activity. Our results demonstrate that CRF acting in the EC can facilitate epileptiform activity.

Another unanswered question regarding the mechanisms by which CRF modulates epilepsy was which receptor (CRF_1_ or CRF_2_) is involved in CRF-mediated facilitation of epilepsy. CRF interacts with two CRF receptors: CRF_1_ and CRF_2_. CRF-induced facilitation of epileptiform activity in the EC is mediated by activation of CRF_2_ not CRF_1_ receptors based on the following lines of evidence. First, the immunoreactivity of CRF_2_ not CRF_1_ receptors was detected in the EC suggesting that CRF_2_ not CRF_1_ should mediate the effects of CRF on epilepsy at least in the EC. Second, pretreatment of slices with antagonists for CRF_2_ receptors blocked CRF-mediated facilitation of epileptiform activity whereas application of the antagonists for CRF_1_ receptors had no effects. Third, application of CRF to slices cut from CRF_2_ KO mice failed to increase the frequency of epileptiform activity whereas CRF still exerted robust facilitatory effects on the frequency of epileptiform activity when applied to slices cut from WT mice. Our results have therefore filled a gap for the effects of CRF on epilepsy by demonstrating that CRF-elicited facilitation of epileptiform activity is mediated by CRF_2_ receptors.

Activation of CRF_2_ receptors increases the function of AC resulting in augmentation of cAMP production and subsequent activation of PKA. Another question we have addressed is whether the AC/cAMP/PKA pathway is involved in CRF-induced enhancement of epileptiform activity. We demonstrate that AC and cAMP are fully required but PKA may be partially necessary for CRF-induced facilitation of epileptiform activity based on the following results. First, inhibition of AC by applying MDL 12330A and SQ 22536 completely blocked CRF-induced augmentation of epileptiform activity. Second, elevation of endogenous cAMP level by forskolin and IBMX increased epileptiform activity. Third, inhibition of PKA by KT 5720 and Rp-cAMPS significantly reduced but not completely blocked CRF-induced increases in epileptiform activity. In accordance with our results, tremendous evidence demonstrates that AC/cAMP/PKA pathway plays a facilitatory role in epilepsy [53], [54], [55], [56], [57], [58].

In conclusion, our results demonstrate that the EC expresses both CRF protein and CRF_2_ receptors and activation of CRF_2_ receptors in the EC facilitates PTX-induced epileptiform activity. CRF-mediated augmentation of epileptiform activity is mediated by CRF_2_-induced increases in intracellular cAMP level and PKA is partially required for its effect on epilepsy.
